The article "Chemical Profiles and Antiobesity Effect of a Mixture of Astragalus membranaceus and Lithospermum erythrorhizon Extract in High Fat Diet Fed Mice" was published in 2022. Journal: Evid Based Complement Alternat Med.

# Chemical Profiles and Antiobesity Effect of a Mixture of *Astragalus membranaceus* and *Lithospermum erythrorhizon* Extract in High Fat Diet Fed Mice

**DOI:** 10.1155/2022/9642427

**Published:** 2022-08-12

**Authors:** Doo Jin Choi, Bo-Ram Choi, HaeJin Lee, Seong Cheol Kim, Dahye Yoon, Young-Seob Lee, Kyung-Sook Han, Sung-Bum Park, Geum-Soog Kim, Dae Young Lee

**Affiliations:** ^1^Department of Herbal Crop Research, National Institute of Horticultural and Herbal Science, RDA, Eumseong 27709, Republic of Korea; ^2^DONG IL Pharm Tec Co. Ltd., Gangnam, Seoul 06296, Republic of Korea; ^3^Department of Biotechnology, The Catholic University of Korea, Bucheon 14662, Republic of Korea

## Abstract

The present study aimed to evaluate the antiobesity potential and synergistic effects of ALM16, a mixture of *Astragalus membranaceus* (AM) and *Lithospermum erythrorhizon* (LE) extracts, in HFD-induced obese mice. C57BL/6 mice were fed a normal diet (ND), high-fat diet (HFD), HFD + AM, HFD + LE or HFD + ALM16 (50, 100, and 200 mg/kg) daily for 5 weeks. Compared to the ND group, HFD-fed mice showed significant increases in body weight, food efficiency ratio, weights of white adipose tissues, adipocytes size, liver weight, and hepatic steatosis grade. However, ALM16 significantly reduced those increases induced by HFD. Moreover, as compared to the HFD group, the ALM16 group significantly ameliorated serum levels of lipid profiles (TG, TC, HDL, and LDL), adipokines (leptin and adiponectin), and liver damage markers (AST and ALT levels). Notably, ALM16 was more effective than AM or LE alone and had a similar or more potent effect than *Garcinia cambogia* extracts, as a positive control, at the same dose. These results demonstrate that ALM16 synergistically exerts anti-obesity effects based on complementary interactions between each component. Also, metabolic profiling between each extract and the ALM16 was confirmed by UPLC-QTOF/MS, and the difference was confirmed by relative quantification.

## 1. Introduction

Obesity is a multifactorial chronic disease characterized by an excess accumulation of fat in adipose tissue due to disturbing the balance between caloric intake and energy expenditure [1, 2]. The World Health Organization (WHO) standards classified the degree of obesity as a body mass index (BMI, weight in kg divided by height squared m^2^). Overweight is defined as having a BMI between 25 and 30 and obesity when BMI exceeds 30 [3]. The prevalence of obesity has increased dramatically worldwide owing to lifestyle and diet changes and is rapidly becoming a major health problem. Obesity not only impacts the status of health itself, but it can also influence to the development of metabolic diseases including type 2 diabetes (T2D), cardiovascular disease, and non-alcoholic fatty liver disease (NAFLD) [4, 5].

The article "Chemical Profiles and Antiobesity Effect of a Mixture of Astragalus membranaceus and Lithospermum erythrorhizon Extract in High Fat Diet Fed Mice" was published in 2022. Journal: Evid Based Complement Alternat Med.

Current therapeutic strategies for obesity are the administration of pharmacological agents including orlistat and sibutramine with the management of diet, exercise, and weight loss [6]. Anti-obesity drugs, mainly synthetic chemicals, are generally known that act as central appetite suppressants, digestion and absorption blockers, metabolic promoters, and obesity gene product inhibitors, however, administration in a long term can cause several adverse effects [7, 8]. For that reason, it is required to develop natural materials with few side effects for obesity management, and herbal medications and functional foods have garnered much attention as potential alternative treatments [9, 10]. Recently herbal medications and natural products, such as raw or extracted products isolated from plants, were reported that they may exert potential health benefits for the treatment of many chronic or complex diseases, including obesity [11]. These herbal products are commonly used as a combination of multiple herbs because they can mediate multi-targets and enhance efficacy or decrease side effects through complementary interactions among individual components [12, 13]. Therefore, extensive studies have been conducted to evaluate various combinations of medicinal herbs as alternative treatments for obesity [14, 15].

*Astragalus membranaceus* (AM), called Hwangki in Korea, is one of the most popular medicinal herbs in traditional medicine in Asia and is extensively used to treat hypertension, diabetes, and many other medical symptoms [16, 17]. AM is well known that can exert various pharmacological properties, including anti-inflammatory, hepatoprotective and neuroprotective effects, containing bioactive constituents such as isoflavonoids, triterpene saponins, and some trace elements [18, 19].

*Lithospermum erythrorhizon* (LE) is extensively used in traditional herbal medicine for the treatment of sore throat and burns, and in traditional distilled liquor, called Jindo Hongju, in Korea [20]. LE is known to contain various phytochemicals such as naphthoquinone pigments and phenolic compounds [21], and is reported to exert antiviral, anti-inflammatory, and antidiabetic activities [22–24]. Numerous studies reported that AM and LE can exert synergistic actions when mixed with other herbs and can be potent complementary herbs [25, 26].

Numerous components have been isolated and reported from AM and LE. Calycosin, formononetin, ononin, and calycosin-7-O-*β*-d-glucoside are representative isoflavonoids isolated from AM. These isoflavonoids are considered bioactive components of AM, and studies on the activity of these components have also been reported including anti-tumor, anti-obesity, and anti-inflammatory [27–29]. In addition, saponins isolated from AM including Astragaloside I-IV are known to have pharmacological effects such as neuroprotective effects, anti-tumor, and anti-obesity [30–32]. In recent research on LE, studies on phenolic compounds such as lithospermic acid and salvianolic acid as well as shikonin have been reported that these chemicals have positive effects on anti-HIV, Parkinson's disease, vascular protection, and antidiabetic effect [33–36].

The article "Chemical Profiles and Antiobesity Effect of a Mixture of Astragalus membranaceus and Lithospermum erythrorhizon Extract in High Fat Diet Fed Mice" was published in 2022. Journal: Evid Based Complement Alternat Med.

In a recent study, we demonstrated that a mixture of two herbal extracts, called ALM16 as a novel formulation, had a hepatoprotective effect against non-alcoholic fatty liver disease (NAFLD) using a mouse model [37]. ALM16 administration significantly inhibited hepatic steatosis in NAFLD mice by modulating AMP-activated protein kinase (AMPK) and acetyl-CoA carboxylase (ACC) signaling pathway in the liver and was more effective than the individual extracts. These observations indicate that ALM16 can exert a synergistic effect, as well as expect a potent biological effect against obesity or metabolic diseases. Although these two herbs have the potential to improve effects mixed with other herbs, the anti-obesity effect of these two herbs combination is poorly explored. Based on this point, the present study aims to evaluate whether ALM16 has an anti-obesity effect in a high-fat diet (HFD)-induced obese mouse model and synergistically enhances the effect over the use of individual herb alone. For comparison, *Garciniacambogia* extract (GC) was used as a positive control in this experiment because it is known to contain hydroxycitric acid (HCA), which inhibits lipogenesis [38]. In addition, simultaneous analysis using UPLC-QTOF/MS was utilized to profile metabolites of each extract for quality control.

## 2. Materials and Methods

### 2.1. UPLC-Q-TOF/MS Analyses

Analysis of compounds in the AMLE mixture was performed using UPLC with Q-TOF/MS. UPLC was performed using a Waters ACUITY H-CLASS UPLC (Waters Corp.,) The mobile phases were composed of solvent A (water and 0.1% formic acid (v/v)) and solvent B (MeCN and 0.1% formic acid (v/v)). The flow rate was 350 *μ*L/min, and the injection volume was 2 *μ*L. The elution conditions were as follows: 0–3.5 min, B 10–35%; 3.5–7 min, B 35–45%; 7–14 min, B 45–95%; 14–16 min, B 95–100; 16–17 min, B 100–100%; 17–18 min, B 100–10%. The column oven and sample tray were maintained at 35°C and 4°C, respectively. MS analysis was carried out using a Waters Xevo G2-S QTOF MS (Waters Corp.,) in negative mode. The mass parameters were set as follows: cone voltage 40 V; capillary 3.0 kV; source temperature 120°C; desolvation temperature 300°C; cone gas flow 30 L/h; and desolvation gas flow 800 L/h. Data were collected between 100 and 2000 m/z using the MSE acquisition mode. An internal reference (Leucine-enkephalin, m/z 554.262 (ESI-)) was used to obtain accurate mass measurements.

The article "Chemical Profiles and Antiobesity Effect of a Mixture of Astragalus membranaceus and Lithospermum erythrorhizon Extract in High Fat Diet Fed Mice" was published in 2022. Journal: Evid Based Complement Alternat Med.

### 2.2. Preparation of ALM16 with AM and LE Extracts

The ALM16 was prepared that the AM and LE extracts were mixed in a ratio of 7 : 3 (w/w), as described in a previous study [39]. The AM (MPS005087) and LE (MPS004961) were purchased from Jecheon, Chungcheongbuk-do, Korea. Briefly, the AM and LE were extracted twice with 50% and 70% aqueous fermented ethanol at 80°C for 4 h, respectively, and the resulting extracts were concentrated, sterilized, dried under pressure (−0.08 MPa), and mixed to produce the ALM16. The powdered samples were stored at −20°C and dissolved in phosphate-buffered saline (PBS) for the in vitro and in vivo experiments.

### 2.3. Animal

Five-week-old C57BL/6 male mice (weighing approximately 16–19 g) were purchased from the ORIENT BIO INC (Gyeonggi-do, Korea), and were housed in the specific pathogen-free (SPF) facility. All mice were treated in accordance with the Guide for the Care and Use of Laboratory Animals, as approved by the Institutional Animal Care and Use Committee of the INVIVO, Co., Ltd. (IACUC proved number, IV-RA-04-1904-05), and all efforts have been made to minimize the number of animals used. During the experiment, mice were maintained under a 12/12-h light-dark cycle at controlled temperatures (22 ± 2°C) and 50 ± 10% humidity for adaptation.

### 2.4. Experiment Design and Treatment

After the acclimatization period, a total of 48 male C57BL/6 mice were randomly allocated into eight groups (6 mice/group): (1) ND: Normal diet (10% Kcal fat), (2) HFD: High-fat diet (60% Kcal fat), (3) AM: HFD + 100 mg/kg *Astragalus membranaceus* extract, (4) LE: HFD + 100 mg/kg *Lithospermum erythrorhizon* extract, (5–7) ALM16-L, M, and H: HFD + 50, 100, and 200 mg/kg mixture of *Astragalus membranaceus* and*Lithospermum erythrorhizon* extracts, respectively, and (8) GC: HFD + 100 mg/kg *Garcinia cambogia* extract (as a positive control). The ND (Cat No. D12350 J) and HFD (Cat No. D12492) were purchased from Research diets, INC. (New Brunswick, NJ, USA). The nutrition facts of the experimental diet are listed in Table 1. After 6 weeks of HFD-induced obesity, all samples were dissolved in PBS and orally administered daily for 5 weeks. The groups fed with ND or HFD only were given an equal volume of PBS by orally administered at the same time. The body weights and food intake of the mice were measured every week. At the end of the experimental period, all mice were fasted for 12 h and were then anesthetized with 2–2.5% isoflurane in oxygen. Blood samples were collected by cardiac puncture. After blood samples were clotted, serum was separated by centrifugation (3,000 rpm, 10 min). Subsequently, white adipose tissues (WATs)—which contain peri-renal (pWAT), retroperitoneal (rWAT), and epididymal (eWAT) —and liver were then collected and weighed. All the processes of the animal experiment were described in Figure 1.

The article "Chemical Profiles and Antiobesity Effect of a Mixture of Astragalus membranaceus and Lithospermum erythrorhizon Extract in High Fat Diet Fed Mice" was published in 2022. Journal: Evid Based Complement Alternat Med.

### 2.5. Serum Biochemical Analysis

Serum levels of triglyceride (TG), total cholesterol (TC), high-density lipoprotein-cholesterol (HDL), and low-density lipoprotein-cholesterol (LDL), as well as aspartate aminotransferase (AST) and alanine aminotransferase (ALT), were measured Automated Biochemistry Analyzer (BS220, Mindray, China). Additionally, commercial enzyme-linked immunosorbent assay (ELISA) kits were used to measure serum levels of leptin (Abcam, Cambridge, UK) and adiponectin (R&D systems, Minneapolis, MN, USA).

### 2.6. Histological Analysis

Liver and eWAT were fixed in 10% formalin and embedded in paraffin. Sections were cut at 3-*μ*m thickness. For histological analysis, sections were stained with hematoxylin and eosin (H&E). Adipocyte size of the eWAT was quantified using a light microscope (Olympus BX50, Olympus Optical Co., Japan). Liver tissue was also examined the hepatic steatosis by a toxicologic pathologist in a blinded manner.

### 2.7. Statistical Analysis

All data are expressed as mean ± standard errors (SE). Statistical analyses were performed with a one-way analysis of variance (ANOVA) followed by Duncan's multiple comparison test using SPSS ver. 12 (SPSS Inc., Chicago, IL, USA). Significant differences between the groups were considered statistically significant when *p* < 0.05. The various components analyzed in ALM16 are shown in Table 2.

## 3. Results

### 3.1. ALM16 Reduced Body Weight and Food Efficiency in HFD-Induced Obese Mice

At the end of the experiment, the HFD group significantly increased (*p* < 0.05) total body weight (40.91 ± 1.75) and body weight gain (25.99 ± 1.14) compared with the ND group (29.85 ± 0.46 g, 11.62 ± 0.46 g). In contrast to the HFD group, ALM16 (100 and 200 mg/kg) administration significantly suppressed total body weight (8.4 and 10.4%, respectively, *p* < 0.05, Figure 2(a)) and body weight gain (26.7 and 28.8%, respectively, *p* < 0.05, Figure 2(b)). Notably, the effects of 100 mg/kg ALM16 on body weight gain were significantly greater than in AM or LE (100 mg/kg) groups, while were similar to the GC (100 mg/kg) group. Food intake did not differ significantly among all experimental groups (Figure 2(c)). The food efficiency ratio (FER) was significantly higher in the HFD group than those of the ND group but decreased in mice treated with AM (*p* > 0.05), LE (*p* < 0.05), ALM16-L (*p* > 0.05), ALM16-M (*p* < 0.05), ALM16-H (*p* < 0.05), or GC (*p* < 0.05) by 9.8, 16.0, 7.3, 15.8, 19.7, or 12.0%, respectively, compared with the HFD group (Figure 2(d)). The administration of 100 and 200 mg/kg of ALM16 was observed to be more potent in body weight gain and FER inhibitory effects than the other groups, but there were no significant differences between these two groups.

The article "Chemical Profiles and Antiobesity Effect of a Mixture of Astragalus membranaceus and Lithospermum erythrorhizon Extract in High Fat Diet Fed Mice" was published in 2022. Journal: Evid Based Complement Alternat Med.

### 3.2. ALM16 Aameliorated Serum Lipid Profiles in HFD-Induced Obese Mice

The serum lipid levels (TG, TC, HDL, and LDL) in the experimental groups were shown in Figure 3. The HFD group increased serum levels of TG (*p* > 0.05, Figure 3(a)), TC (*p* < 0.05, Figure 3(b)), LDL (*p* < 0.05, Figure 3(d)) by 9.4, 9.4, and 8.6%, respectively, compared to the ND group, but decreased serum levels of HDL (*p* > 0.05, Figure 3(c)). In contrast, the ALM16 (100 mg/kg) group significantly reduced (*p* < 0.05) the serum levels of TG, TC, and LDL by 18.9, 17.5, and 29.0%, respectively, compared to the HFD group, while significantly increased (*p* < 0.05) serum levels of HDL by 18.7%. ALM16 (100 mg/kg) group was shown to be similar to or more effective on the serum levels of lipid than the other doses of ALM16 groups. The LE group had significantly decreased the serum levels of TG (*p* < 0.05) by 9.4%, whereas it had no significant differences in the serum levels of TC, LDL, and HDL compared to the HFD group. In addition, the AM group had no significant differences in the serum levels of TG, TC, HDL, and LDL compared to the HFD group.

### 3.3. ALM16 Ameliorated Adipokine Levels in HFD-Induced Obese Mice

Serum leptin levels of HFD-fed mice (37,198.2 ± 4,475.9 pg/ml) significantly increased (*p* < 0.05) by 18.6-fold compared to the ND group (1,997.6 ± 302.9 pg/ml). However, AM, LE, ALM16-L, M, H, and GC groups decreased the serum leptin levels by 8.2, 22.4, 13.4, 29.5, 21.1, and 19.0% respectively, compared with the HFD group. Interestingly, serum leptin levels in the ALM16-M group (*p* < 0.05) were significantly lower than in the HFD group and were more effective when compared to AM, LE, and GC at the same dose (Figure 4(a)). The serum adiponectin levels of the ND group (19,231.9 ± 213.6 ng/ml) were significantly higher than in the HFD group (17,494 ± 351.6 ng/ml, *p* < 0.05). However, the decrease of serum adiponectin levels induced by HFD was significantly increased in the AM, LE, ALM16-L, M, H, and GC groups by 7.1, 6.3, 8.2, 10.5, 7.2, and 10.2%, respectively, compared to the HFD group (Figure 4(b)). Interestingly, administration of ALM16 (100 mg/kg) was more effective than administration of AM or LE (100 mg/kg) alone. The ALM16-M (19337.7 ± 86.6 ng/ml) and GC (19281.9 ± 166.3 ng/ml) groups had increased serum adiponectin levels similar to the ND group.

The article "Chemical Profiles and Antiobesity Effect of a Mixture of Astragalus membranaceus and Lithospermum erythrorhizon Extract in High Fat Diet Fed Mice" was published in 2022. Journal: Evid Based Complement Alternat Med.

### 3.4. ALM16 Suppressed Fat Accumulation of White Adipose Tissues in HFD-Induced Obese Mice

To investigate the effects of ALM16 on weights and masses of WATs in HFD-induced obese mice, the weights and masses of WATs were monitored at the end of the experiment. As shown in Figure 5(a), the masses of pWAT, rWAT, and eWAT were higher in the HFD group than in the ND group, respectively. However, all treated groups showed reduced masses of WATs compared with the HFD group. The weights of WATs were significantly increased in the HFD group compared to the ND group (*p* < 0.05, Figure 5(b)–5(d)). ALM16 100 mg/kg group showed significantly reduced weights of pWAT, rWAT, and eWAT by 23.1, 15.6, and 44.5%, respectively, compared with the HFD group (*p* < 0.05). Interestingly, the weight of eWAT showed a significant reduction effect in the ALM16 (100 mg/kg) than in the GC (100 mg/kg) group. In addition, AM and LE groups had no significant differences in the weights of pWAT and eWAT, respectively, compared to the HFD group, but had a significant inhibitory effect on the rWAT weight gain. Adipocyte size in eWAT was examined in H&E stained sections. The adipocyte size was significantly larger in the HFD group than in the ND group (*p* < 0.05, Figure 6(a)), whereas it was significantly smaller in the AM, LE, ALM16 (L, M, and H) groups (*p* < 0.05, respectively) than in the HFD group (Figure 6(b)).

### 3.5. ALM16 Inhibited Hepatic Steatosis and Liver Damage in HFD-Induced Obese Mice

Histological changes and weight gain in the liver tissues of the experimental groups were shown in Figure 7. The liver section of the HFD group observed a severe accumulation of lipid droplets compared to that of the ND group which appeared as clear (Figure 7(a)), as well as was significantly higher hepatic steatosis grade (2.50 ± 0.22, *p* < 0.05) than in the ND group (0.17 ± 0.17, Figure 7(b)). In addition, the HFD group exhibited a significant increase in liver weight (1.62 ± 0.16, *p* < 0.05) compared with the ND group (1.01 ± 0.02, Figure 7(c)). In contrast, administration of ALM16 (L, M, and H) and GC significantly reduced the deposition of lipids in the liver tissue, hepatic steatosis grade (1.50 ± 0.22, 1.00 ± 0.00, 1.00 ± 0.00, and 1.00 ± 0.26, respectively, *p* < 0.05), and liver weights (1.23 ± 0.05, 1.09 ± 0.04, 1.13 ± 0.05, and 1.10 ± 0.03 g, respectively, *p* < 0.05) compared to the those of the HFD group. In the AM and LE groups, although no significant effects on hepatic steatosis were observed, the liver weight gains were significantly inhibited by the administration of AM (1.33 ± 0.08 g) or LE (1.21 ± 0.08 g) compared to the HFD group. Moreover, the HFD group showed significantly higher serum levels of AST and ALT (as the markers of liver damage), respectively, when compared to that of the ND group (*p* < 0.05, Figure 7(d) and 7(e)). However, the ALM16 (100 mg/kg) group showed significant reductions (19.4 and 49.8% reduction, respectively) in both serum levels of AST and ALT compared with the HFD group. The inhibitory effects of ALM16 (100 mg/kg) on serum levels of AST and ALT were more potent than those of the AM or LE group.

The article "Chemical Profiles and Antiobesity Effect of a Mixture of Astragalus membranaceus and Lithospermum erythrorhizon Extract in High Fat Diet Fed Mice" was published in 2022. Journal: Evid Based Complement Alternat Med.

### 3.6. Profiling and Quantification of Various Components from ALM16 Using UPLC-QTOF/MS

UPLC-QTOF/MS with an in-house library was conducted to profile the metabolites in ALM16, AM, and LE extracts. The total ion chromatograms (TICs) of ALM16, AM, and LE extracts were shown in Figure 8. The intensities of major peaks in AM extracts were decreased in ALM16. The major peaks of LE extracts also showed this decrease in the ALM16. The decrease in the major peak of the LE extracts in ALM16 was more pronounced than in AM extracts, probably because the proportion of LE extracts was lower in the ALM16. The peak intensities were analyzed for the relative quantification of ALM16, AM, and LE extracts and confirmed metabolic change. For relative quantification analysis, eight kinds of *Astragalus membranaceus* derived components including calycosin and calycosin-7-O-*β*-D-glucoside and lithospermic acid and salvianolic acid A, which are components derived from *Lithospermum erythrorhizon* were analyzed using the in-house library. In the relative quantification of ALM16, the intensity of AM-derived components such as calycosin and astragaloside was decreased similarly to the mixture ration, and lithospermic acid and salvianolic acid A, which are LE-derived components, also decreased in the AML16.

## 4. Discussion

Obesity is a complex and chronic disease characterized by excessive accumulation of lipids. Obesity represents a severe health problem worldwide because it can increase the risk of many metabolic diseases such as diabetes mellitus, hyperlipidemia, and fatty liver disease [4, 5]. Both AM and LE demonstrated various biological and pharmacological activities, including anti-inflammatory [23, 40] and anti-obesity properties [41, 42], but few studies have reported the obesity and synergistic effects of a mixture of these two herbal extracts. Therefore, the present study aimed to determine whether ALM16, a mixture of AM and LE extracts (7 : 3, w/w), can exert the anti-obesity effect and be more effective than those of individual materials.

The article "Chemical Profiles and Antiobesity Effect of a Mixture of Astragalus membranaceus and Lithospermum erythrorhizon Extract in High Fat Diet Fed Mice" was published in 2022. Journal: Evid Based Complement Alternat Med.

Our previous study reported that ALM16 contains three compounds (calycosin-7-O-*β*-D-glucoside, calycosin, and lithospermic acid, as chemical markers), and exerts a chondroprotective effect in an osteoarthritis rat model, based on synergistic actions [40]. In addition, in the previous study, only three representative compounds of ALM16 were identified, but in this study, UPLC-QTOF/MS profiling was performed on ALM16 to analyze the components of a mixture. Through profiling analysis, ten components including three compounds previously studied were identified in the mixture. Various components identified through analysis are known to have various physiological activities including anti-obesity and related activities. In a previous study using an in vitro obesity model, ononin showed anti-adipogenic capacity by upregulating SIRT1 and inhibiting PI3K, PPAR*γ,* and adiponectin [43]. In addition, astragaloside IV is known to prevent obesity in a high-fat diet mouse model [32] and is also known to have a positive effect on obesity-related nephropathy and hypertension [44, 45]. Obesity is caused by the expansion of white adipose tissue and a decrease in brown adipose tissue. In a previous study by Lai et al., salvianolic acid A increased browning of white adipose tissue in high-fat diet-induced mice [46]. It is thought that components such as ononin or salvianolic acid may have affected the anti-obesity activity of the ALM16 in various ways. Herbal mixtures are expected to play multiple synergistic roles than single extracts. Therefore, it is necessary to identify and confirm the various components in the mixture.

The ALM16 was selected effective ratio of 7 : 3 (w/w) by screening the chondroprotective effect among combinations mixed with the different ratios at in vitro model [47]. In recent, many studies have focused on identifying the novel combination of diverse herbs that possess beneficial effects for the treatment of multifactorial and chronic diseases [48, 49]. This is because the combination materials can exert multifunctional and multi-targeting through complementary interactions between each component according to the combination and mixing ratio of herbs. In our previous study, we further investigated and reported the hepatoprotective effect of ALM16 on hepatic steatosis in a non-alcoholic fatty liver disease (NAFLD) rodent model, indicating that ALM16 may have multifunctional properties [37]. Since the development of NAFLD is directly associated with obesity, we hypothesized that ALM16, which has confirmed protective effects against NAFLD, may have anti-obesity activity.

The article "Chemical Profiles and Antiobesity Effect of a Mixture of Astragalus membranaceus and Lithospermum erythrorhizon Extract in High Fat Diet Fed Mice" was published in 2022. Journal: Evid Based Complement Alternat Med.

For this purpose, we investigated the anti-obesity effect of AM, LE, and ALM16 using the HFD-induced obese mice model, which is the most widely used in obesity studies, as it closely resembles abnormalities parallelling the progression of human obesity [50]. In addition, it is well known that HFD feeding in rodents can readily induce obesity conditions such as increases in body weight gain, mass and weight of white adipose tissues, and levels of lipid profiles [51]. The result of this study showed that these parameters, which indicate obesity status, were significantly increased in the HFD group compared to the ND group. However, ALM16 effectively inhibited the increase in parameters induced by HFD feeding and was more effective than individual extract administrations. Zheng et al. reported that a combination of Erigeron annuus L. Pers and Borago officinalis L. was a markedly more potent anti-obesity effect than alone due to synergistic actions of certain functional components [52]. Han et al. reported that calycosin in AM directly improves perivascular adipose tissue dysfunction in obese mice [53]. Gwon et al. reported that LE has an anti-obesity effect by suppressing adipogenic transcriptional factors in white adipose tissue and is partially attributed to acetyl shikonin [42]. Consequently, our results indicated that ALM16 can synergistically exert anti-obesity effects, although understanding of the cross interactions between individual components is required.

Leptin is one of the adipokines that is primarily secreted from adipose tissue and is involved in the increase of BMI and adipose tissue mass through the regulation of appetite and energy expenditure [54]. Koh et al. reported that HFD feeding in rodent models increases serum leptin levels, contributing to increased weight gain and fat accumulation [3]. In addition, adiponectin is one of the adipokines secreted by adipocytes to control glucose and lipid metabolism, and energy homeostasis in both humans and animals [55]. A number of anti-obesity studies have reported that serum adiponectin levels are decreased by HFD feeding, while elevated serum adiponectin levels are associated with a reduction in body weight gain [56,57]. It is well known that adiponectin in the liver activates fatty acid oxidation through the peroxisome proliferator-activated receptor *α* (PPAR*α*) pathway and regulates fat lipid metabolism [58]. In various studies for anti-obesity treatment, increased adiponectin expression has been accepted as a major target, which has demonstrated therapeutic benefits in animal models [59, 60]. Therefore, the serum levels of leptin and adiponectin can be considered representative parameters of the obesity state. Similar to tendencies of previous studies, our results showed that ALM16 inhibited the increase in serum leptin levels by HFD feeding while increasing the reduced serum adiponectin levels. Hence, these results indicate that ALM16 may exert a positive effect on body weight gain, FER, fat mass, and WATs weight through regulation of serum adipokines levels. White adipose tissue (WAT) is an energy storage site and secret adipokines such as leptin and adiponectin [61]. WAT, which increases the size and number of adipocytes due to excessive fat accumulation in the obese state, leads to dysregulation of adipokines expression and causes related metabolic abnormalities [62].

The article "Chemical Profiles and Antiobesity Effect of a Mixture of Astragalus membranaceus and Lithospermum erythrorhizon Extract in High Fat Diet Fed Mice" was published in 2022. Journal: Evid Based Complement Alternat Med.

The liver is known as a key tissue that plays an important role in lipid metabolism including hepatic lipogenesis and fatty acid oxidation [63]. Various studies have observed elevated liver weight gain, hepatic steatosis condition, and liver toxicity induced by excessive hepatic lipid accumulation in rodents fed an HFD [64, 65]. Similarly, our results showed that the HFD group increased liver weight, hepatic steatosis grade, and serum levels AST and ALT associated with signs of liver damage, while the ALM16 group effectively ameliorated that fatty liver state. Thus, these results provide potent evidence that ALM16 may also exert a beneficial effect against hepatic steatosis, which is closely associated with dietary obesity.

Meanwhile, the present study may provide scientific evidence to assess clinical effectiveness in the future but it has some limitations. First of all, the experiment was investigated with a small sample size, therefore, further study of large sample size is needed. Second, we investigated using the mice's limited conditions such as same sexual and certain age. To objectify, the additional approach using mice in various conditions is also required.

## 5. Conclusions

The present study demonstrated that ALM16 reduced weights of body and white adipose tissues, serum levels of lipid profiles, and adipokines in HFD-induced obese mice. In addition, ALM16 ameliorated HFD-induced increases in liver weight, hepatic steatosis, and liver damage. In particular, ALM16 showed more potent activity against obesity in mice fed HFD than individual extracts. These results suggest that ALM16 synergistically has the anti-obesity and anti-hepatic steatosis effects, and ultimately exerts multifunctional properties. Therefore, ALM16 may be considered a potential material for anti-obesity functional foods.

## Figures and Tables

**Figure 1:** Overall process of animal experiment.

The article "Chemical Profiles and Antiobesity Effect of a Mixture of Astragalus membranaceus and Lithospermum erythrorhizon Extract in High Fat Diet Fed Mice" was published in 2022. Journal: Evid Based Complement Alternat Med.

**Figure 2:** Effects of ALM16 on body weight and food intake in HFD-fed mice; (a) changes in body weight, (b) body weight gain, (c) food intake, and (d) food efficiency ratio (FER). Data are expressed as mean ± SE (*n* = 6). Different letters indicate statistical differences between groups at *p* < 0.05. ND: Normal diet; HFD: High-fat diet; AM: HFD + 100 mg/kg AM extract; LE: HFD + 100 mg/kg LE extract; ALM16-L: 50 mg/kg ALM16; ALM16-M: 100 mg/kg ALM16; ALM16-H: HFD + 200 mg/kg ALM16; GC: HFD + 100 mg/kg GC extract.

**Figure 3:** Effects of ALM16 on serum lipid profiles in HFD-induced obese mice; (a) serum levels of triglyceride (TG), (b) total cholesterol (TC), (c) HDL-cholesterol, and (d) LDL-cholesterol in HFD-fed mice. Data are expressed as mean ± SE (*n* = 6). Different letters indicate statistical differences between groups at *p* < 0.05. ND: Normal diet; HFD: High-fat diet; AM: HFD + 100 mg/kg AM extract; LE: HFD + 100 mg/kg LE extract; ALM16-L: 50 mg/kg ALM16; ALM16-M: 100 mg/kg ALM16; ALM16-H: HFD + 200 mg/kg ALM16; GC: HFD + 100 mg/kg GC extract.

**Figure 4:** Effects of ALM16 on adipokines production in HFD-induced obese mice; (a) serum levels of leptin and (b) adiponectininHFD-fed mice were measured by ELISA assay. Data are expressed as mean ± SE (*n* = 6). Different letters indicate statistical differences between groups at *p* < 0.05. ND: Normal diet; HFD: High-fat diet; AM: HFD + 100 mg/kg AM extract; LE: HFD + 100 mg/kg LE extract; ALM16-L: 50 mg/kg ALM16; ALM16-M: 100 mg/kg ALM16; ALM16-H: HFD + 200 mg/kg ALM16; GC: HFD + 100 mg/kg GC extract.

**Figure 5:** Inhibitory effects of ALM16 on weight gain of white adipose tissues (WATs) gain in HFD-induced mice; (a) photographs of representative WATs, (b) weights of peri-renal WAT, (c) retroperitoneal WAT, and (d) epididymal WAT from mice fed an HFD. Data are expressed as mean ± SE (*n* = 6). Different letters indicate statistical differences between groups at *p* < 0.05. ND: Normal diet; HFD: High-fat diet; AM: HFD + 100 mg/kg AM extract; LE: HFD + 100 mg/kg LE extract; ALM16-L: 50 mg/kg ALM16; ALM16-M: 100 mg/kg ALM16; ALM16-H: HFD + 200 mg/kg ALM16; GC: HFD + 100 mg/kg GC extract.

**Figure 6:** Effect of ALM16 on lipid accumulation in epididymal white adipose tissue (eWAT) in HFD-induced obese mice; (a) representative histological images of H&E stained eWAT (magnification, 4×, scale bar 100 *μ*m) and (b) adipocytes size were quantified under microscope. Data are expressed as mean ± SE (*n* = 6). Different letters indicate statistical differences between groups at *p* < 0.05. ND: normal diet; HFD: high-fat diet; AM: HFD + 100 mg/kg AM extract; LE: HFD + 100 mg/kg LE extract; ALM16-L: 50 mg/kg ALM16; ALM16-M: 100 mg/kg ALM16; ALM16-H: HFD + 200 mg/kg ALM16; GC: HFD + 100 mg/kg GC extract.

The article "Chemical Profiles and Antiobesity Effect of a Mixture of Astragalus membranaceus and Lithospermum erythrorhizon Extract in High Fat Diet Fed Mice" was published in 2022. Journal: Evid Based Complement Alternat Med.

**Figure 7:** Protective effects of ALM16 against hepatic steatosis and liver damage in HFD-induced obese mice; (a) representative histological images of the liver were assessed using H&E staining (magnification, 4×, scale bar 100 *μ*m),(b) steatosis grade and (c) weight of liver in HFD-induced obese mice, (d) Serum levels of ALT, and (e) AST in HFD-induced obese mice. Data are expressed as mean ± SE (*n* = 6). Different letters indicate statistical differences between groups at *p* < 0.05. ND: normal diet; HFD: high-fat diet; AM: HFD + 100 mg/kg AM extract; LE: HFD + 100 mg/kg LE extract; ALM16-L: 50 mg/kg ALM16; ALM16-M: 100 mg/kg ALM16; ALM16-H: HFD + 200 mg/kg ALM16; GC: HFD + 100 mg/kg GC extract.

**Figure 8:** The total ion chromatograms of (a) AM extracts, (b) LE extracts, and (c) ALM16.

**Table 1:** Composition of experimental diet.

Components	Normal diet		High-fat diet	
	gm%	Kcal%	gm%	Kcal%
Protein	19.2	20	26.2	20
Carbohydrate	67.3	70	26.3	20
Fat	4.3	10	34.9	60
Total		100		100
Ingredient	gm	Kcal	gm	Kcal
Casein, 30 mesh	200	800	200	800
L-Cystine	3	12	3	12
Corn starch	506.2	2024.8	0	0
Maltodextrin 10	125	500	125	500
Sucrose	68.8	275.2	68.8	275.2
Cellulose, BW200	50	0	50	0
Soybean oil	25	225	25	225
Lard	20	180	245	2205
Mineral Mix S10026	10	0	10	0
DiCalcium phosphate	13	0	13	0
Calcium carbonate	5.5	0	5.5	0
Potassium citrate	16.5	0	16.5	0
Vitamin Mix V10001	10	40	10	40
Choline bitartrate	2	0	2	0
FD&C yellow dye #5	0.04	0	—	—
FD&C blue dye #5	0.01	0	0.05	0
Total	1055.05	4057	773.85	4057

**Table 2:** The list of various components analyzed in ALM16.

No.	Components	RT (min)	Molecular formula	Expected neutral mass (Da)	Observed neutral mass (Da)	Observed m/z	Mass error (ppm)	Relative quantification (mg/g)
1	Calycosin-7-O-*β*-D-glucoside	2.45	C_22_H_22_O_10_	446.1213	446.1211	491.1193	−0.4	0.5
2	Lithospermic acid	3.21	C_27_H_22_O_12_	538.1113	538.1101	537.1029	−1.8	0.3
3	Ononin	3.6	C_22_H_22_O_9_	430.1263	430.1259	475.1241	−1.1	0.35
4	Salvianolic acid A	3.7	C_26_H_22_O_10_	494.1213	494.1209	439.1136	−0.8	2.112
5	Calycosin	3.99	C_16_H_12_O_5_	284.0684	284.0678	283.0605	−2.5	0.479
6	Astragaloside IV	5.45	C_41_H_68_O_14_	784.4609	784.4617	829.4599	1	0.487
7	Formononetin	5.58	C_16_H_12_O_4_	268.0735	268.0732	267.066	−1.2	0.659
8	Astragaloside III	5.6	C_41_H_68_O_14_	784.4609	784.4619	829.4601	1.3	0.891
9	Astragaloside II	6.3	C_43_H_70_O_15_	826.4714	826.4723	871.4705	1	1.404
10	Astragaloside I	8.08	C_45_H_72_O_16_	868.482	868.483	913.4814	1.2	1.411

## Data Availability

The datasets used and/or analyzed during the current study are available from the corresponding author on reasonable request.

The article "Chemical Profiles and Antiobesity Effect of a Mixture of Astragalus membranaceus and Lithospermum erythrorhizon Extract in High Fat Diet Fed Mice" was published in 2022. Journal: Evid Based Complement Alternat Med.

## References

[1] Romieu I., Dossus L., Barquera S. (2017). Energy balance and obesity: what are the main drivers?. *Cancer Causes & Control*.

[2] Spiegelman B. M., Flier J. S. (2001). Obesity and the regulation of energy balance. *Cell*.

[3] Koh Y. M., Jang S. W., Ahn T. W. (2019). Anti-obesity effect of Yangkyuksanwha-tang in high-fat diet-induced obese mice. *BMC Complementary and Alternative Medicine*.

[4] Scherer P. E., Hill J. A. (2016). Obesity, diabetes, and cardiovascular diseases: a compendium. *Circulation Research*.

[5] Fabbrini E., Sullivan S., Klein S. (2010). Obesity and nonalcoholic fatty liver disease: biochemical, metabolic and clinical implications. *Hepatology*.

[6] Pilitsi E., Farr O. M., Polyzos S. A. (2019). Pharmacotherapy of obesity: available medications and drugs under investigation. *Metabolism*.

[7] Apovian C. M., Aronne L. J., Bessesen D. H. (2015). Pharmacological management of obesity: an endocrine society clinical practice guideline. *Journal of Clinical Endocrinology and Metabolism*.

[8] Torgerson J. S., Hauptman J., Boldrin M. N., Sjöström L. (2004). XENical in the prevention of diabetes in obese subjects (XENDOS) study: a randomized study of orlistat as an adjunct to lifestyle changes for the prevention of type 2 diabetes in obese patients. *Clinical Diabetology*.

[9] Hasani-Ranjbar S., Larijani B., Abdollahi M. (2009). A systematic review of the potential herbal sources of future drugs effective in oxidant-related diseases. *Inflammation and Allergy—Drug Targets*.

[10] Hasani-Ranjbar S., Nayebi N., Moradi L., Mehri A., Larijani B., Abdollahi M. (2010). The efficacy and safety of herbal medicines used in the treatment of hyperlipidemia; a systematic review. *Current Pharmaceutical Design*.

[11] Chien M. Y., Ku Y. H., Chang J. M., Yang C. M., Chen C. H. (2016). Effects of herbal mixture extracts on obesity in rats fed a high-fat diet. *Journal of Food and Drug Analysis*.

[12] Williamson E. M. (2001). Synergy and other interactions in phytomedicines. *Phytomedicine*.

[13] Yang Y., Zhang Z., Li S., Ye X., Li X., He K. (2014). Synergy effects of herb extracts: pharmacokinetics and pharmacodynamic basis. *Fitoterapia*.

[14] Kim D. S., Kim S. H., Cha J. (2016). Antiobesity effects of the combined plant extracts varying the combination ratio of Phyllostachys pubescens leaf extract and Scutellaria baicalensis root extract. *Evidence-based Complementary and Alternative Medicine*.

[15] Sim W. S., Choi S. I., Cho B. Y. (2019). Anti-obesity effect of extract from *Nelumbo nucifera* L., *morus alba* L., and *raphanus sativus* mixture in 3T3-L1 adipocytes and C57BL/6J obese mice. *Foods*.

The article "Chemical Profiles and Antiobesity Effect of a Mixture of Astragalus membranaceus and Lithospermum erythrorhizon Extract in High Fat Diet Fed Mice" was published in 2022. Journal: Evid Based Complement Alternat Med.

[16] Zhang J. Q., Xie X. S., Li C., Fu P. (2009). Systematic review of the renal protective effect of *Astragalus membranaceus* (root) on diabetic nephropathy in animal models. *Journal of Ethnopharmacology*.

[17] Gui S. Y., Wei W., Wang H. (2006). Effects and mechanisms of crude astragalosides fraction on liver fibrosis in rats. *Journal of Ethnopharmacology*.

[18] He X., Shu J., Xu L., Lu C., Lu A. (2012). Inhibitory effect of Astragalus polysaccharides on lipopolysaccharide-induced TNF-a and IL-1*β* production in THP-1 cells. *Molecules*.

[19] Fu J., Wang Z., Huang L. (2014). Review of the botanical characteristics, phytochemistry, and pharmacology of *Astragalus membranaceus* (huangqi). *Phytotherapy Research*.

[20] Chen X., Yang L., Oppenheim J. J., Howard O. M. Z. (2002). Cellular pharmacology studies of shikonin derivatives. *Phytotherapy Research*.

[21] Choi Y. H., Kim G. S., Choi J. H. (2016). Ethanol extract of *Lithospermum erythrorhizon*Sieb. et Zucc. promotes osteoblastogenesis through the regulation of Runx2 and Osterix. *International Journal of Molecular Medicine*.

[22] Zhang Y., Han H., Sun L. (2017). Antiviral activity of shikonin ester derivative PMM-034 against enterovirus 71 in vitro. *Brazilian Journal of Medical and Biological Research*.

[23] Yoshida L. S., Kakegawa T., Yuda Y., Takano-Ohmuro H. (2017). Shikonin changes the lipopolysaccharide-induced expression of inflammation-related genes in macrophages. *Journal of Natural Medicines*.

[24] Öberg A. I., Yassin K., Csikasz R. I. (2011). Shikonin increases glucose uptake in skeletal muscle cells and improves plasma glucose levels in diabetic Goto-Kakizaki rats. *PLoS One*.

[25] Zhou X., Seto S. W., Chang D. (2016). Synergistic effects of Chinese herbal medicine: a comprehensive review of methodology and current research. *Frontiers in Pharmacology*.

[26] Roh J. S., Lee H., Lim J. (2017). Effect of Gangjihwan on hepatic steatosis and inflammation in high fat diet-fed mice. *Journal of Ethnopharmacology*.

[27] Huang C., Li R., Shi W., Huang Z. (2019). Discovery of the anti-tumor mechanism of calycosin against colorectal cancer by using system pharmacology approach. *Medical Science Monitor*.

[28] Nie T., Zhao S., Mao L. (2018). The natural compound, formononetin, extracted from Astragalus membranaceus increases adipocyte thermogenesis by modulating PPAR*γ* activity. *British Journal of Pharmacology*.

[29] Dong L., Yin L., Chen R. (2018). Anti-inflammatory effect of Calycosin glycoside on lipopolysaccharide-induced inflammatory responses in RAW 264.7 cells. *Gene*.

[30] Luo Y., Qin Z., Hong Z. (2004). Astragaloside IV protects against ischemic brain injury in a murine model of transient focal ischemia. *Neuroscience Letters*.

The article "Chemical Profiles and Antiobesity Effect of a Mixture of Astragalus membranaceus and Lithospermum erythrorhizon Extract in High Fat Diet Fed Mice" was published in 2022. Journal: Evid Based Complement Alternat Med.

[31] Chen X., Chen X., Gao J. (2019). Astragaloside III enhances anti-tumor response of NK cells by elevating NKG2D and IFN-*γ*. *Frontiers in pharmacology*.

[32] Wu H., Gao Y., Shi H. L. (2016). Astragaloside IV improves lipid metabolism in obese mice by alleviation of leptin resistance and regulation of thermogenic network. *Scientific Reports*.

[33] Varadaraju T. G., Hwu J. R. (2012). Synthesis of anti-HIV lithospermic acid by two diverse strategies. *Organic and Biomolecular Chemistry*.

[34] Lin Y. L., Tsay H. J., Lai T. H., Tzeng T. T., Shiao Y. J. (2015). Lithospermic acid attenuates 1-methyl-4-phenylpyridine-induced neurotoxicity by blocking neuronal apoptotic and neuroinflammatory pathways. *Journal of Biomedical Science*.

[35] Wu Y., Xu S., Tian X. Y. (2020). The effect of salvianolic acid on vascular protection and possible mechanisms. *Oxidative Medicine and Cellular Longevity*.

[36] Qiang G., Yang X., Shi L. (2015). Antidiabetic effect of salvianolic acid A on diabetic animal models via AMPK activation and mitochondrial regulation. *Cellular Physiology and Biochemistry*.

[37] Choi D. J., Kim S. C., Park G. E. (2020). Protective effect of a mixture of *Astragalus membranaceus* and *Lithospermum erythrorhizons* extract against hepatic steatosis in high fat diet-induced nonalcoholic fatty liver disease mice. *Evidence-based Complementary and Alternative Medicine*.

[38] Mvaia-Landim A., Ramírez J. M., Lancho C., Poblador M. S., Lancho J. L. (2018). Long-term effects of Garcinia *cambogia*/Glucomannan on weight loss in people with obesity, PLIN4, FTO and Trp64Arg polymorphisms. *BMC Complementary and Alternative Medicine*.

[39] Choi D. J., Choi S. I., Choi B. R., Lee Y. S., Lee D. Y., Kim G. S. (2019). Cartilage protective and anti-analgesic effects of ALM16 on monosodium iodoacetate induced osteoarthritis in rats. *BMC Complementary and Alternative Medicine*.

[40] Su X., Huang Q., Chen J. (2016). Calycosin suppresses expression of pro-inflammatory cytokines *via* the activation of p62/Nrf2-linked heme oxygenase 1 in rheumatoid arthritis synovial fibroblasts. *Pharmacological Research*.

[41] Huang Y. C., Tsay H. J., Lu M. K. (2017). Astragalus membranaceusAstragalus membranaceus-polysaccharides ameliorates obesity, hepatic steatosis, neuroinflammation and cognition impairment without affecting amyloid deposition in metabolically stressed APPswe/PS1dE9 mice. *International Journal of Molecular Sciences*.

[42] Gwon S. Y., Ahn J. Y., Chung C. H., Moon B., Ha T. Y. (2012). *Lithospermum erythrorhizon* suppresses high-fat diet-induced obesity, and acetylshikonin, a main compound of *lithospermum erythrorhizon*, inhibits adipocyte differentiation. *Journal of Agricultural and Food Chemistry*.

The article "Chemical Profiles and Antiobesity Effect of a Mixture of Astragalus membranaceus and Lithospermum erythrorhizon Extract in High Fat Diet Fed Mice" was published in 2022. Journal: Evid Based Complement Alternat Med.

[43] Mladenova S. G., Savova M. S., Marchev A. S. (2022). Anti-adipogenic activity of maackiain and ononin is mediated via inhibition of PPAR*γ* in human adipocytes. *Biomedicine & Pharmacotherapy*.

[44] Li Z., Yang W., Yang Y., Wu J., Luo P., Liu Y. (2022). The Astragaloside IV derivative LS-102 ameliorates obesity-related nephropathy. *Drug Design, Development and Therapy*.

[45] Jiang P., Ma D., Wang X. (2018). Astragaloside IV prevents obesity-associated hypertension by improving pro-inflammatory reaction and leptin resistance. *Molecules and Cells*.

[46] Lai J., Qian Q., Ding Q. (2021). Activation of AMP-activated protein kinase-sirtuin 1 pathway contributes to salvianolic acid a-induced browning of white adipose tissue in high-fat diet fed male mice. *Frontiers in Pharmacology*.

[47] Choi D. J., Choi B. R., Lee D. Y., Choi S. I., Lee Y. S., Kim G. S. (2019). Inhibitory effect of mixed extracts obtained from Astragali radix and Lithospermi radix on matrix metalloproteinases in IL-1*β*-induced SW1353 cells and quantitative analysis of active compounds. *Korean Journal of Medicinal Crop Science*.

[48] Lee D., Ju M. K., Kim H. (2020). Commiphora extract mixture ameliorates monosodium iodoacetate-induced osteoarthritis. *Nutrients*.

[49] Cho B. O., Choi J., Kang H. J. (2020). Anti-obesity effects of a mixed extract containing *Platycodon grandiflorum, Apium graveolens* and green tea in high-fat-diet-induced obese mice.Platycodon grandiflorum, *Apium graveolens* and green tea in high-fat-diet-induced obese mice. *Experimental and Therapeutic Medicine*.

[50] Kanasaki K., Koya D. (2011). Biology of obesity: lessons from animal models of obesity. *Journal of Biomedicine and Biotechnology*.

[51] Hariri N., Thibault L. (2010). High-fat diet-induced obesity in animal models. *Nutrition Research Reviews*.

[52] Zheng Y., Lee J., Shin K. O., Park K., Kang I. J. (2019). Synergistic action of *Erigeron annuus L*. Pers and *Borago officinalis* L. enhances anti-obesity activity in a mouse model of diet-induced obesity. *Nutrition Research*.

[53] Han F., Li K., Pan R. (2018). Calycosin directly improves perivascular adipose tissue dysfunction by upregulating the adiponectin/AMPK/eNOS pathway in obese mice. *Food & Function*.

[54] Elmquist J. K. (2000). Anatomic basis of leptin action in the hypothalamus. *Frontiers of Hormone Research*.

[55] Meier U., Gressner A. M. (2004). Endocrine regulation of energy metabolism: review of pathobiochemical and clinical chemical aspects of leptin, ghrelin, adiponectin, and resistin. *Clinical Chemistry*.

The article "Chemical Profiles and Antiobesity Effect of a Mixture of Astragalus membranaceus and Lithospermum erythrorhizon Extract in High Fat Diet Fed Mice" was published in 2022. Journal: Evid Based Complement Alternat Med.

[56] Hsu C. H., Tsai T. H., Kao Y. H., Hwang K. C., Tseng T. Y., Chou P. (2008). Effect of green tea extract on obese women: a randomized, double-blind, placebo-controlled clinical trial. *Clinical Nutrition*.

[57] Rahman H. A., Sahib N. G., Saari N. (2017). Anti-obesity effect of ethanolic extract from *Cosmos caudatus*Kunth leaf in lean rats fed a high fat diet. *BMC Complementary and Alternative Medicine*.

[58] Nigro E., Scudiero O., Monaco M. L. (2014). New insight into adiponectin role in obesity and obesity-related diseases. *BioMed Research International*.

[59] Yamazaki Y., Kawano Y., Uebayasi M. (2008). Induction of adiponectin by natural and synthetic phenolamides in mouse and human preadipocytes and its enhancement by docosahexaenoic acid. *Life Sciences*.

[60] Sahebkar A. (2013). Head-to-head comparison of fibrates versus statins for elevation of circulating adiponectin concentrations: a systematic review and meta-analysis. *Metabolism*.

[61] Longo M., Zatterale F., Naderi J. (2019). Adipose tissue dysfunction as determinant of obesity-associated metabolic complications. *International Journal of Molecular Sciences*.

[62] Zorena K., Jachimowicz-Duda O., Ślęzak D., Robakowska M., Mrugacz M. (2020). Adipokines and obesity. Potential link to metabolic disorders and chronic complications. *International Journal of Molecular Sciences*.

[63] Huh J. H., Kim K. J., Kim S. U. (2017). Obesity is more closely related with hepatic steatosis and fibrosis measured by transient elastography than metabolic health status. *Metabolism*.

[64] Park Y. J., Lee G. S., Cheon S. Y., Cha Y. Y., An H. J. (2019). The anti-obesity effects of Tongbi-san in a high-fat diet-induced obese mouse model. *BMC Complementary and Alternative Medicine*.

[65] Sung Y. Y., Kim D. S., Kim S. H., Kim H. K. (2018). Aqueous and ethanolic extracts of Welsh onion, *Allium fistulosum*, attenuate high-fat diet-induced obesity. *BMC Complementary and Alternative Medicine*.

